# Association of Hyperhomocysteinemia with Increased Coronary Microcirculatory Resistance and Poor Short-Term Prognosis of Patients with Acute Myocardial Infarction after Elective Percutaneous Coronary Intervention

**DOI:** 10.1155/2020/1710452

**Published:** 2020-01-02

**Authors:** Yang-Pei Peng, Ming-Yuan Huang, Yang-Jing Xue, Jia-Lin Pan, Cong Lin

**Affiliations:** Department of Cardiology, The Second Affiliated Hospital of Wenzhou Medical University, Wenzhou, Zhejiang 325000, China

## Abstract

**Background:**

This study aims to investigate the coronary microcirculatory resistance and prognosis of patients with acute myocardial infarction (AMI) concomitant with hyperhomocysteinemia (HHcy) after an elective percutaneous coronary intervention (PCI).

**Methods:**

A total of 101 patients that underwent elective PCI between May 2015 and July 2018 due to AMI were consecutively enrolled in this study. Patients were divided into a HHcy group (53) and a normal Hcy group (control; 48) based on their plasma homocysteine concentration. The characteristics of coronary angiography, the index of microcirculatory resistance (IMR) of infarct-related vessels (IRV), changes in left ventricular end diastolic diameter (LVEDd) and left ventricular ejection fraction (LVEF) before and after PCI, and the incidence of major adverse cardiovascular events (MACE) three months after PCI were compared between these groups.

**Results:**

Compared to the results from the Hcy group, the HHcy group had a higher IMR. The HHcy group had significantly higher LVEDd and a lower LVEF than the Hcy group 3 months after PCI. Additionally, the incidence of MACE at three months after PCI was higher in the HHcy group than in the Hcy group. Pearson correlation analysis revealed a positive correlation with IMR in the HHcy group. Furthermore, there was a difference in the LVEDd measured at one day after PCI and at three months after PCI in the HHcy group.

**Conclusion:**

AMI patients concomitant with HHcy that undergo elective PCI are prone to coronary microcirculatory dysfunction and have a poor cardiac function and poor prognosis at three months after PCI.

## 1. Introduction

Acute myocardial infarction (AMI) is one of the most common cardiac diseases worldwide and has three clinical forms: acute non-ST-segment elevation myocardial infarction (NSTEMI), ST-segment elevation myocardial infarction (STEMI), and unstable angina [1]. While it has been well recognized that AMI is caused by a blockade of the coronary arteries, coronary microcirculation, which is essential for the survival of the local myocardium and myocardial recovery after AMI [2], also plays an important role in disease development, progression, and prognosis. Indeed, several studies have revealed that impaired microcirculation predicts the poor outcomes of AMI patients [3, 4]. Currently, the mainstay of treatment for patients with AMI is percutaneous coronary intervention (PCI). However, PCI may also cause microcirculatory dysfunction, thus, leading to a poor prognosis [5]. Hence, an accurate determination of the functional status of the microcirculation offers a valuable assessment of the outcomes of patients with AMI after PCI. Among these measures, the index of microcirculatory resistance (IMR) is a relatively simple quantitative measure of coronary microcirculatory function and is considered to be a reliable indicator of the extent of coronary vascular bed expansion. For instance, Fearon et al. found that the IMR obtained immediately after emergency PCI in STEMI patients was significantly negatively correlated with the postoperative echocardiographic wall motion scores obtained three months after PCI, as evidenced by the observation that the group with an IMR >32 had a significantly lower wall motion score than that of the group with an IMR <32 [6]. Additionally, they proposed that an IMR >40 is a predictor of death or hospitalization due to heart failure [7], and an elevated IMR after AMI has been shown to be an important indicator of a lowered myocardial survival rate [8]. Therefore, IMR is an appropriate index for the evaluation of microcirculatory function in AMI patients.

Homocysteine (Hcy) is an amino acid that is generated through protein breakdown. A high plasma Hcy level, hyperhomocysteinemia (HHcy), plays an important role in arterial damage and thrombosis [9]. Recent studies have shown that HHcy contributes to a high IMR and circulating hs-CRP in patients with coronary atherosclerotic stenosis [10]. Furthermore, HHcy is an independent predictor of increased coronary microcirculation resistance [10]. Additionally, HHcy is closely associated with an increased risk of long-term adverse events in patients with coronary artery diseases [11]. Moreover, the long-term risk of all-cause mortality of patients that have undergone PCI is significantly higher when plasma Hcy levels exceed 13.5 *μ*mol/L [12]. Together, these findings suggest that there is a prognostic value of HHcy in patients with cardiac diseases. However, whether HHcy may be used to predict the outcomes of patients with AMI that have undergone elective PCI has not been well explored. This study aimed to investigate whether the coronary microcirculatory resistance, as reflected by IMR, could be used to assess the short-term prognosis of patients with AMI complicated by HHcy.

## 2. Materials and Methods

### 2.1. Ethics Statement

This study protocol was approved by the Ethics Committee of the Second Affiliated Hospital of Wenzhou Medical University. Written informed consent was obtained from all participants.

### 2.2. Subject Selection

A total of 101 patients that were undergoing elective PCI due to acute NSTEMI or STEMI in the Second Hospital affiliated to Wenzhou Medical University between May 2017 and May 2019 were consecutively selected for this study. Patients who had acute occlusion of at least one major epicardial coronary artery were included in this study. None of the patients had accepted the thrombolytic therapy. Patients who had one or more of the following traits were excluded from our study: (1) uncontrolled severe heart failure (ejection fraction < 35%), (2) inability to tolerate dual antiplatelet therapy, (3) extremely slow arrhythmia (hearty rate < 50/min), (4) hemorrhagic disease, (5) asthma or severe pulmonary dysfunction, (6) a history of coronary artery bypass surgery, (7) severe liver and kidney dysfunction, and (8) acute and chronic infectious diseases. Based on a cut-off plasma Hcy level of 10 *μ*mol/L defined by the American Heart Association (AHA) [13] before PCI, these patients were divided into two groups: a HHcy group (Hcy > 10 *μ*mol/L; *n* = 53) and a normal Hcy group (control; Hcy < 10 *μ*mol/L; *n* = 48).

The diagnostic criteria for hypercholesterolemia were based on the following recommendations for the prevention and treatment of dyslipidemia that were formulated in 1997 in China: total cholesterol (TC) > 5.2 mmol/L, low-density lipoprotein cholesterol > 3.4 mmol/L, or plasma TC concentration after adequate lipid-lowering therapy was controlled. Diabetes mellitus was diagnosed based on the following criteria, defined by the American Diabetes Association: fasting blood glucose >7.0 mmol/L or insulin injection and/or the requirement of hypoglycemic drugs to maintain blood glucose within the normal range. Hypertension was diagnosed based on the Joint National Committee VII (JNC VII) guidelines: systolic blood pressure (SBP) > 140 mmHg and/or diastolic blood pressure (DBP) > 90 mmHg, or the patient had a history of chronic hypertension and needed oral antihypertensive drugs to control the blood pressure. Smoking was referred to as a continuous period of smoking that lasted more than six months. A high BMI was defined as a BMI >24 kg/m^2^. Chronic kidney disease was defined as a glomerular filtration rate lower than 60 ml/min/1.73 m^2^ or a positive marker of renal injury without a decrease in glomerular filtration rate.

### 2.3. Elective PCI

All patients underwent coronary angiography and balloon dilatation and stenting for infarct-related vessels (IRV). A successful stent was defined as having all of the following features: significant relief or disappearance of chest pain, a fully expanded and adherent stent as revealed by angiography, less than 20% of the residual stenosis of the target vessel, no intimal tear or dissection, and a thrombolysis in myocardial infarction (TIMI) grade III flow.

### 2.4. Determination of IMR

IMR was obtained using pressure and temperature sensitive guidewire (St. Jude Medical Company, Sweden) after stent implantation of all IRVs. The procedure is briefly described as follows: (1) aortic pressure was set to zero and the guidewire was calibrated outside of the body; (2) the guidewire was sent to the guide catheter port to calibrate the pressure and temperature, and the pressure of the ostium of the guidewire was equalized to the pressure of the ostium of the guide catheter, which was similar to the mean aortic pressure (Pa) and was used as a pressure reference. Additionally, the corrected temperature was used as a reference for subsequent temperature changes; (3) the guidewire was further pushed through the lesion segment and exceeded two-thirds of the total length; (4) intracoronary nitroglycerin (200 *μ*g) was injected to minimize the coronary arterial tone; (5) three milliliters of room temperature normal saline was quickly injected using the thermal dilution technique. When the liquid entered the ostium of the coronary artery, the pressure guide shaft recorded the first temperature curve. When the liquid passed through the sensor of the head of the guidewire, the second temperature curve was recorded. The time difference between the recording of the first and the second temperature curve was defined as the mean transit time (Tmn). The mean transit time of the baseline (bTmn) was obtained from three continuous measurements; (6) ATP (140 *μ*g/kg/min, over 3–6 min) was pumped through the elbow vein to maximize hyperemia of the coronary artery, followed by rapid injection of 3 ml of normal saline after 90 seconds three times in a row to obtain the mean transit time under hyperemia (hTmn); (7) the Pa values at the resting and hyperemic state and the mean distal coronary pressure (Pd) at the stenotic lesion were recorded, and the IMR was calculated by the machine based on the following formula: IMR = Pd × Tmn.

### 2.5. Plasma Hcy Measurement

Two days before angiography, a 5 ml blood sample was collected from an elbow vein of each patient. This sample was placed in a test tube containing ethylenediaminetetraacetic acid and centrifuged at 2,500 rpm/min for 20 minutes. The supernatant was collected and stored at −20°C. The plasma Hcy concentration was measured using an ELISA kit (DADE Behring, USA) and a Biochemical Automated Analyzer (DADE Behring, USA).

### 2.6. Follow-Up

Echocardiography was performed for all patients using an ultrasound system (IE33, Philips) at one day and three months after PCI. The examination conditions were as follows: the probe frequency was 2.0 MHz∼4.0 MHz and the Doppler velocity range was −30 cm/s∼30 cm/s. Several important cardiac functional parameters, including left ventricular end diastolic diameter (LVEDd) and left ventricular ejection fraction (LVEF), were recorded. The LVEF was measured using the Simpson biplane method. At three months after PCI, major adverse cardiovascular events (MACE) were defined as the occurrence of cardiac death, recurrent myocardial infarction and angina pectoris, severe heart failure, malignant arrhythmia, and retargeted revascularization, as previously reported [14].

### 2.7. Statistical Analysis

All statistical analyses were performed using SPSS 20.0 software (USA). Measurement data are expressed as mean ± standard deviation (SD). After the Kolmogorov–Smirnov test for normality, comparisons were calculated using *t*-tests and analysis of variance (ANOVA) between groups, while the *X*^2^ test was used to compare the count data. Linear regression analysis was used to examine the correlation between the Hcy concentration and IMR and the changes in LVEDd and LVEF of each patient between one day and three months after PCI. Pearson correlation analysis and multivariate logistic regression analysis were used to evaluate the relationship between total MACE and the related risk factors at 3 months after PCI. Statistical significance was defined as a *P* value less than 0.05.

## 3. Results

### 3.1. Comparison of the Demographic and Basal Clinical Characteristics of Patients between the Two Groups

As shown in Table 1, there were no significant differences in the age, smoking habits, BMI, hypertension, hyperlipidemia, diabetes, chronic kidney disease, PCI, or common biochemical test results and medications between the HHcy and control groups (*P* > 0.05). As expected, the plasma Hcy concentration was significantly higher in the HHcy group than in the control group (14.15 ± 3.30 mmol/L vs. 6.67 ± 1.66 mmol/L, *P* < 0.01). Additionally, the hs-CRP level was higher in the HHcy group than in the control group (10.9 ± 1.3 mg/L vs. 9.7 ± 1.6 mg/L, *P* < 0.01).

### 3.2. Comparison of Coronary Angiographic Characteristics and IMR between the Two Groups

We next evaluated the differences in the coronary angiographic characteristics and IMR between the HHcy group and the control group. As shown in Table 2, there were no statistically significant differences in the number of diseased coronary arteries, the TIMI flow grades, the morphological characteristics of the atherosclerotic lesions, or the intracoronary distribution between the two groups (*P* > 0.05). Additionally, no difference was observed in the vascular sites between the two groups, as evaluated by pressure guidewire (*P* > 0.05). However, the IMR was significantly higher in the HHcy group than in the control group (*P* < 0.01).

### 3.3. Comparison of Cardiac Function and the Incidence of MACE after PCI between the Two Groups

The differences in LVEDd and LVEF were not statistically significant between the HHcy group and the control group at one day after PCI (*P* > 0.05). However, the LVEDd was significantly higher in the HHcy group than in the control group (52.3 ± 4.2 mm vs. 48.4 ± 4.6 mm, *P* < 0.01) 3 months after PCI. Furthermore, the difference in the LVEDd between one day and three months after PCI was significantly higher in the HHcy group than in the control group (4.2 ± 2.0 mm vs. 1.1 ± 2.5 mm, *P* < 0.01). At three months after PCI, the LVEF was significantly lower in the HHcy group than in the control group (47.8 ± 6.4% vs. 54.7 ± 6.1%, *P* < 0.01). Additionally, the difference in the LVEF between one day and three months after PCI was significantly lower in the HHcy group than in the control group (−2.2 ± 2.8% vs. 2.6 ± 2.9%, *P* < 0.01). We also found that the incidence of MACE was significantly higher in the HHcy group than in the control group 3 months after PCI (24.5% vs. 6.3%, *P*=0.019; Table 3).

### 3.4. Determination of Risk Factors for MACE Three Months after PCI

Univariate linear regression and logistic regression analysis showed that Hcy, LVEF, and age were independent risk factors for MACE three months after PCI in patients with AMI, with correlation coefficients (*r*) of 0.324, 0.389, and 0.304 and odds ratios of 3.741, 4.986, and 2.652, respectively. Among these risk factors, LVEF had the strongest correlation with MACE, followed by Hcy (Table 4).

### 3.5. Correlation between Hcy and IMR and Changes in LVEDd and LVEF

The correlations between the level of Hcy with IMR and the changes in LVEDd and LVEF between one day and three months after PCI were determined using Pearson correlation analysis and multivariate logistic regression analysis. The Hcy level was positively correlated with the IMR (*r* = 0.502, *P* < 0.01) and the LVEDd change between one day and three months after PCI (*r* = 0.421, *P* < 0.01). However, the Hcy level was negatively correlated with the LVEF change (*r* = –0.536, *P* < 0.01; Figure 1 and Table 5).

## 4. Discussion

In the present study, we evaluated the coronary microcirculatory resistance and short-term prognosis of patients with AMI complicated by HHcy. We found that (1) there was a positive correlation between HHcy and the IMR and LVEDd changes between one day and three months after PCI, (2) there was a negative correlation between HHcy and LVEF changes between one day and three months after PCI, and (3) HHcy was an independent factor for MACEs in patients with AMI after selective PCI. Our study provides a strong rationale for effectively controlling the plasma Hcy levels of patients with AMI before performing the PCI procedure. There are also views that high Hcy was only a concomitant factor of coronary heart disease, and intervention of Hcy did not reduce the risk of cardiovascular and cerebrovascular diseases [15, 16]. The reasons accounting for some findings that treatment of HHcy did improve the prognosis may be attributed to many factors, including a multifactorial disease, age, gender, hypertension, hyperlipidemia, elevated serum creatinine, coffee and alcohol intake, and folic acid and vitamin B12 intake, which may all affect Hcy levels. Therefore, these interfering factors may have effects on the above findings to some degree.

Previous studies have shown that there is a link between the plasma Hcy level and cardiovascular diseases and that this is considered to be an independent predictor of the outcome in patients with AMI. For instance, elevated circulating Hcy levels are associated with increased mortality and overall adverse outcomes of patients with AMI even after successful coronary angioplasty [17]. Additionally, the inclusion of plasma Hcy levels in the Framingham Coronary Heart Disease Risk Score System substantially increases the predictive value of the risk of coronary heart disease and risk of cardiovascular events [18]. Therefore, it has been proposed that Hcy serves as a modifiable cardiovascular risk factor and holds a predictive value for the severity of cardiovascular diseases [19–21]. In line with the above findings, in the present study, we also found a positive correlation between HHcy and MACEs in patients with AMI after PCI. Together, these findings point to the importance of lowering the plasma Hcy in patients with AMI.

In the present study, we found that the IMR was significantly higher in the HHcy group than in the control group. Additionally, we found that the level of Hcy was positively correlated with the IMR, suggesting that patients with AMI with HHcy were prone to more severe coronary microcirculatory dysfunction. No significant differences in LVEDd and LVEF were observed between the two groups on the first day after PCI. This suggests that the patients in both groups had comparable cardiac function prior to PCI. However, three months after PCI, the LVEDd and LVEDd differences were significantly higher and the LVEF changes between one day and three months after PCI were significantly lower in the HHcy group than in the group with normal plasma Hcy levels. These observations indicate that the cardiac function is more severely impaired following selective PCI in AMI patients with HHcy, as evidenced by the observation of elevated circulating hs-CRP levels in AMI patients with HHcy. Although HHcy and elevated hs-CRP were independent risk factors of cardiovascular diseases [22] and the combination of these two features improved the predictive value of the outcome of cerebrovascular diseases [23], it was not clear whether there was any correlation between HHcy and elevated hs-CRP levels. Because hs-CRP is an indicator of an inflammatory response, our findings suggest that HHcy potentially exacerbates AMI-induced inflammation in the heart. Collectively, these findings suggest that the recovery of cardiac function in AMI patients with HHcy three months after PCI was not as good as that observed in control patients. Therefore, we believe that AMI patients with HHcy that miss emergency PCI have a poorer prognosis than those without HHcy, even if they undergo elective PCI at a later date.

Traditional and nontraditional risk factors for coronary heart disease can damage the endothelial function of epicardial vessels and distal microvessels, which may cause endothelial cell-dependent dysfunction, especially in patients with AMI [24]. While PCI has been shown to efficiently restore the blood flow to the infarcted region of the heart, it also increases the epicardial vascular endothelial dysfunction and promotes thrombus detachment, subsequently leading to an increased risk of distal microcirculatory embolization, which in turn results in decreased myocardial perfusion and compromised postoperative rehabilitation in patients with AMI [25]. Several studies have demonstrated that an elevated Hcy level is an independent risk factor for coronary endothelial cell dysfunction [26, 27]. Indeed, the level of plasma Hcy affects the body's coagulation function by injuring vascular endothelial cells, causing inflammatory responses of arterial blood vessels [28]. The present study also revealed that the level of hs-CRP was significantly elevated in the HHcy group. A previous study [29] found that HHcy inhibits the repair of myocardial cells after MI. The main mechanisms through which this occurs are the suppression of stem cell factor-induced repair and increased myocardial interstitial fibrosis, leading to thickening, hardening, and hyaline degeneration of the arteriolar wall. However, several prospective clinical trials have reported no significant correlation between HHcy and atherothrombotic vascular disease [30]. Whether there is a close correlation between HHcy and cardiovascular diseases and whether the lowering of plasma Hcy levels would be clinically helpful remain to be clarified in future studies.

This study had some limitations. For example, this was a single-center retrospective study with a small sample size. Thus, the findings of this study should be further corroborated in large cohort studies in the future. Additionally, this study did not include any investigations into the effect of preangiography medications on the IMR.

In conclusion, we report that HHcy is positively correlated with the IMR and the severity of cardiac dysfunction, and also serves as a prognostic factor for MACEs in patients with AMI after selective PCI.

## Figures and Tables

**Figure 1:** Correlation between the homocysteine levels and index of microcirculatory resistance (IMR) (a), the differences in the left ventricular ejection fraction (LVEDd) (b), and the left ventricular ejection fraction (LVEF) (c) between one day and three months after selective PCI of patients.

**Table 1:** Comparison of the demographic and basal clinical characteristics of patients between the two groups.

Characteristics	HHcy group (*n* = 53)	Control group (*n* = 48)	*P*	*X* ^2^ (*t*)
Age (years)	57.3 ± 10.9	55.9 ± 8.8	0.500	0.677
Gender, male (%)	30 (56.6%)	25 (47.2%)	0.649	0.208
BMI (kg/m^2^)	27.3 ± 3.2	27.0 ± 4.0	0.696	0.391
CKD	7 (13.2%)	4 (7.5%)	0.432	0.617
Smoker	23 (43.4%)	16 (30.2%)	0.300	1.076
Hypertension	21 (39.6%)	18 (34.0%)	0.827	0.048
Diabetes mellitus	19 (35.8%)	16 (30.2%)	0.791	0.070
Dyslipidemia	24 (45.3%)	22 (45.8%)	0.956	0.003
Previous PCI	17 (32.1%)	18 (37.5%)	0.567	0.327
STEMI	48 (90.6%)	45 (93.8%)	0.554	0.350
FBG (mmol/L)	6.0 ± 1.2	5.8 ± 9.3	0.479	0.711
Cre (*μ*moI/L)	74.8 ± 15.3	74.6 ± 13.9	0.286	1.072
LDL-C (mmol/L)	3.1 ± 0.5	3.0 ± 0.6	0.228	1.213
HDL-C (mmol/L)	1.4 ± 0.4	1.6 ± 0.5	0.249	−1.161
CTnI (ng/ml)	0.86 ± 0.69	0.71 ± 0.35	0.191	1.316
BNP (pg/ml)	453.6 ± 124.6	393.3 ± 204.9	0.074	1.806
Hs-CRP (mg/L)	10.9 ± 1.3	9.7 ± 1.6	0.000	4.116
Medications:				
Beta-blocker	38 (71.7%)	35 (72.9%)	0.891	0.019
Calcium-blocker	24 (45.3%)	20 (41.7%)	0.714	0.134
Aspirin	53 (100%)	48 (100%)	1.000	
Clopidogrel	53 (100%)	48 (100%)	1.000	
Atorvastatin	51 (96.2%)	47 (97.9%)	0.617	0.250
Nitrates	32 (60.4%)	30 (62.5%)	0.827	0.048
ACEI/ARB	31 (58.5%)	30 (62.5%)	0.681	0.169
Homocysteine (*μ*mol/L)	14.15 ± 3.30	6.67 ± 1.66	0.000	14.152

HHcy: high homocysteine; BMI: body mass index; CKD: chronic kidney diseases; PCI: percutaneous coronary intervention; FBG: fasting blood glucose; LDL-C: low-density lipoprotein cholesterol; HDL-C: high-density lipoprotein cholesterol; CTnI: cardiac troponin I; Hs-CRP: high-sensitivity C-reactive protein; ACEI: angiotensin-converting enzyme inhibitor; ARB: angiotensin receptor blocker.

**Table 2:** Comparison of coronary angiographic characteristics and IMR between the two groups.

		HHcy (*n* = 53)	Control (*n* = 48)	*P*	*X* ^2^ (*t*)
Culprit vessel number	1	31 (58.5%)	23 (47.9%)	0.287	1.132
	2	18 (34.0%)	21 (43.8%)	0.313	1.018
	3	4 (7.5%)	4 (8.3%)	0.884	0.021
TIMI flow grade	0	0	0	1	
	1	0	0	1	
	2	3 (5.7%)	2 (4.2%)	0.730	0.119
	3	50 (94.3%)	46 (95.8%)	0.730	0. 119
Culprit vessel	LMCA	1 (1.9%)	0 (0%)	0.339	0.915
	LAD	37 (67.9%)	32 (64.6%)	0.734	0.115
	Circumflex	6 (11.3%)	5 (10.4%)	0.884	0.021
	RCA	9 (17.0%)	11 (22.9%)	0.455	0.559
Side branch		25 (47.2%)	29 (60.4%)	0.183	1.777
IMR		38.28 ± 8.05	27.13 ± 4.83	0.000	8.336

HHcy: high homocysteine; TIMI: thrombolysis in myocardial infarction; LMCA: left main coronary artery; LAD: left anterior descending artery; RCA: right coronary artery; IMR: index of microvascular resistance.

**Table 3:** Comparison of cardiac function and the incidence of MACE after PCI between the two groups.

		HHcy (*n* = 53)	Control (*n* = 48)	*P*	*X* ^2^ (*t*)
LVEDd (mm)	1^st^ day after PCI	48.2 ± 3.7	47.3 ± 4.6	0.325	0.989
	3 months after PCI	52.3 ± 4.2	48.4 ± 4.6	0.000	4.410
	Difference	4.2 ± 2.0	1.1 ± 2.5	0.000	6.780
EF (%)	1st day after PCI	50.0 ± 7.4	52.1 ± 6.8	0.142	−1.479
	3 months after PCI	47.8 ± 6.4	54.7 ± 6.1	0.000	−5.535
	Difference	−2.2 ± 2.8	2.6 ± 2.9	0.000	−8.573
Total number of MACE		13 (24.5%)	3 (6.3%)	0.019	5.503

HHcy: high homocysteine; LVEDd: left ventricular end diastolic dimension; EF: ejection fraction; MACE: major adverse cardiovascular events.

**Table 4:** Determination of risk factors for MACE at three months after PCI.

	Univariate regression analysis				Logistic regression analysis			
	MACE (*n* = 16)	None-MACE (*n* = 95)	*X* ^2^ (*t*)	*P*	*B*	*r*	OR	*P*
Age	57.5 ± 9.6	52.0 ± 10.8	0.996	0.041	0.769	0.297	2.652	0.031
Male	10 (62.5%)	48 (50.5%)	0.787	0.375				
Smoker	7 (43.8%)	34 (35.8%)	0.373	0.542				
Hypertension	8 (50.0%)	32 (33.7%)	1.314	0.252				
Diabetes mellitus	5 (31.3%)	30 (31.6%)	0.001	0.979				
Dyslipidemia	7 (43.8%)	39 (41.1%)	0.041	0.839				
BMI ≥24 kg/m^2^	9 (56.3%)	51 (53.7%)	0.036	0.849				
CKD	1 (6.3%)	10 (10.5%)	0.280	0.596				
Previous PCI	8 (50.0%)	27 (28.4%)	2.954	0.086				
Calcium-blocker	8 (50.0%)	36 (37.9%)	0.839	0.360				
Beta-blocker	10 (62.5%)	63 (66.3%)	0.089	0.766				
ACEI/ARB	10 (62.5%)	51 (53.7%)	0.430	0.512				
Nitrates	11 (68.8%)	51 (53.7%)	1.261	0.262				
Statins	15 (93.8%)	94 (98.9%)	2.091	0.148				
EF	42.9 ± 5.0	52.5 ± 6.5	5.63	<0.01	0.986	0.389	4.986	0.022
Hcy	15.32 ± 4.93	9.70 ± 3.96	−5.004	<0.01	0.805	0.324	3.741	0.029

MACE: major adverse cardiovascular events. BMI: body mass index; CKD: chronic kidney diseases; PCI: percutaneous coronary intervention; ACEI: angiotensin-converting enzyme inhibitor; ARB: angiotensin receptor blocker; EF: ejection fraction; Hcy: homocysteine.

**Table 5:** Correlation between Hcy and IMR and changes in LVEDd and EF.

	*r*	*P*
IMR	0.502	<0.01
LVEDd difference (mm)	0.421	<0.01
EF difference (%)	–0.536	<0.01

IMR: index of microvascular resistance; LVEDd: left ventricular end diastolic dimension; EF: ejection fraction.

## Data Availability

The data sets generated and analyzed during the current study are available from the corresponding author upon reasonable request.
